The article "Proline-Rich Tyrosine Kinase 2 (Pyk2) Regulates IGF-I-Induced Cell Motility and Invasion of Urothelial Carcinoma Cells" was retracted in 2019. Reason: duplicated images.

# Proline-Rich Tyrosine Kinase 2 (Pyk2) Regulates IGF-I-Induced Cell Motility and Invasion of Urothelial Carcinoma Cells

**DOI:** 10.1371/journal.pone.0040148

**Published:** 2012-06-28

**Authors:** Marco Genua, Shi-Qiong Xu, Simone Buraschi, Stephen C. Peiper, Leonard G. Gomella, Antonino Belfiore, Renato V. Iozzo, Andrea Morrione

**Affiliations:** 1 Endocrine Mechanisms and Hormone Action Program, Department of Urology, Kimmel Cancer Center, Thomas Jefferson University, Philadelphia, Pennsylvania, United States of America; 2 Cancer Cell Biology and Signaling Program, Department of Pathology, Anatomy and Cell Biology, Kimmel Cancer Center, Thomas Jefferson University, Philadelphia, Pennsylvania, United States of America; 3 Endocrinology, Department of Health, University of Catanzaro, Catanzaro, Italy; Aix-Marseille University, France

## Abstract

The insulin-like growth factor receptor I (IGF-IR) plays an essential role in transformation by promoting cell growth and protecting cancer cells from apoptosis. We have recently demonstrated that the IGF-IR is overexpressed in invasive bladder cancer tissues and promotes motility and invasion of urothelial carcinoma cells. These effects require IGF-I-induced Akt- and MAPK-dependent activation of paxillin. The latter co-localizes with focal adhesion kinases (FAK) at dynamic focal adhesions and is critical for promoting motility of urothelial cancer cells. FAK and its homolog Proline-rich tyrosine kinase 2 (Pyk2) modulate paxillin activation; however, their role in regulating IGF-IR-dependent signaling and motility in bladder cancer has not been established. In this study we demonstrate that FAK was not required for IGF-IR-dependent signaling and motility of invasive urothelial carcinoma cells. On the contrary, Pyk2, which was strongly activated by IGF-I, was critical for IGF-IR-dependent motility and invasion and regulated IGF-I-dependent activation of the Akt and MAPK pathways. Using immunofluorescence and AQUA analysis we further discovered that Pyk2 was overexpressed in bladder cancer tissues as compared to normal tissue controls. Significantly, in urothelial carcinoma tissues there was increased Pyk2 localization in the nuclei as compared to normal tissue controls. These results provide the first evidence of a specific Pyk2 activity in regulating IGF-IR-dependent motility and invasion of bladder cancer cells suggesting that Pyk2 and the IGF-IR may play a critical role in the invasive phenotype in urothelial neoplasia. In addition, Pyk2 and the IGF-IR may serve as novel biomarkers with diagnostic and prognostic significance in bladder cancer.

## Introduction

Bladder cancer is a major epidemiological problem, whose incidence continues to rise. The most recent cancer statistic has estimated 73,510 new cases and 14,880 estimated deaths in the United States for 2012 [1]. The majority of bladder tumors (∼70%) are low-grade noninvasive papillary tumors that do not penetrate the epithelial basement membrane (Ta stage). The remainder comprise tumors that have penetrated the basement membrane but not invaded the muscle layer of the bladder wall (T1 stage) and muscle-invasive tumors (T2, T3 and T4 stages) [2], [3], [4]. The prognosis for low-grade tumors is generally good, but about 10%–15% of these patients will later develop invasive disease. For invasive tumors the prognosis is much less favorable, with only 50% survival at 5 years. Invasive tumors frequently progress to life-threatening metastases, which is associated with a 5 year survival rate of 6% [3], [4]. Thus, understanding the mechanisms that regulate bladder tumor invasion is critical to predict and treat this devastating condition in bladder cancer patients.

It is well established that the insulin-like growth factor receptor I (IGF-IR) plays a critical role in cell growth both *in vitro* [5] and *in vivo* [6]. Mice with targeted ablation of the *IGF-IR* gene have severe growth retardation, being only 45% the size of wild-type littermates [7], [8]. Studies performed in mouse embryo fibroblasts derived from the *IGF-IR*-deficient mice (R- cells) have really underscored the essential role of the IGF-IR in transformation [9]. R-cells are indeed refractory to transformation induced by several tumorigenic agents (viral oncogenes such as Ras and SV40 large T Ag, as well as over-expressed PDGFR and EGFR, and various chemical agents) but are transformed upon IGF-IR re-expression [10], [11]. Experiments on tumor cell lines and epidemiological studies have confirmed that activation of the IGF-IR is involved in the development of many common neoplastic diseases, including carcinomas of lung, prostate, pancreas, liver, colon and breast [10], [12], [13]. The transforming capability of the IGF-IR most likely depends on its ability to protect cancer cells from apoptosis [11], [12], [14], [15], [16].

We have recently demonstrated that the IGF-IR is upregulated in invasive and high-grade bladder cancer tumor tissues compared to low-grade and normal tissue controls and promotes motility and invasion of urothelial cancer cells [17], [18]. Significantly, IGF-IR activation did not induce cell proliferation of bladder cancer cells, indicating that the IGF-IR acts as a “scatter factor” for urothelial carcinoma-derived cells and may regulate the transition to the invasive stage of bladder cancer [17]. We also showed that IGF-IR-dependent cell motility and invasion required the activation of the Akt and MAPK pathway [17], [18] and Akt- and ERK-dependent activation of paxillin, which upon IGF-I-stimulation colocalized with focal adhesion kinase (FAK) in dynamic adhesions at the leading edge of migrating urothelial cancer cells and was critical for IGF-I-induced motility of these cells [17].

Here we show that while FAK was not required for IGF-IR-dependent signaling and motility of invasive urothelial carcinoma cells, the FAK-related Pyk2 [19], [20] was strongly activated by IGF-I in urothelial carcinoma cells, was critical for IGF-IR-dependent motility and invasion and regulated IGF-I-dependent activation of the Akt and MAPK pathways. We also discovered that Pyk2 is overexpressed in bladder cancer tissues compared to normal tissue controls and that there is a striking increase in Pyk2 translocation to the nuclei of these malignant cells.

Collectively, these results provide novel information toward a better understanding of the mechanisms that regulate tumor progression in bladder cancer and suggest that Pyk2 and the IGF-IR may be critical for the transition to the invasive phenotype. In addition, these studies could potentially contribute to the identification of novel targets for therapeutic intervention in bladder tumors.

## Results

### FAK Activity in the Regulation of IGF-I-induced Migration, Invasion and Signaling

We recently discovered that paxillin plays an important role in regulating IGF-IR-dependent motility of urothelial carcinomas [17]. It is well established that FAK regulates paxillin activation [21] and the assembly/disassembly of focal adhesions (adhesion turnover) at the cell front of migrating cells [22]. However, it **is** not yet established whether FAK or its homolog Pyk2 [19], [20], which is also expressed by urothelial cancer cells, may play a role in regulating IGF-I-induced motility of bladder cancer cells. Thus, we first employed small interfering RNA (siRNA) strategies to transiently deplete endogenous FAK in 5637 invasive urothelial carcinoma cells and then assessed FAK function in the regulation of IGF-I-induced motility and invasion. We reached a very significant depletion of endogenous FAK with the anti-FAK siRNA (Figure 1A). The oligos were specific for FAK insofar as there was no effect on Pyk2 expression levels (Figure 1A). Notably, FAK depletion did not induce a statistically-significant decrease in IGF-I-mediated migratory response in 5637 cells compared to either parental or scrambled oligos-transfected cells (Figure 1B). However, the invasive ability of 5637 cells was reduced, although at levels barely below statistical significance (P = 0.046) as compared to control oligos-transfected cells (Figure 1C). In addition, using immunoblot analysis with phospho-specific antibodies, we discovered that FAK depletion did not affect IGF-I-mediated activation of the MAPK or Akt pathways (Figure 1D), which are both necessary for IGF-IR-dependent motility and invasion of urothelial cancer cells [17], [18].

**Figure 1:** FAK is not important for IGF-I-mediated motility and signaling of invasive urothelial cancer cells. (A) 5637 cells were transfected with the FAK siGenome pool or control oligos. After 72 hours FAK and Pyk2 expression was detected by immunoblot with specific antibodies. Blot is representative of three independent experiments with an average FAK depletion level of 93.3±3.5 (arbitrary units) as assessed by densitometric analysis (B and C) Migration and invasion assays of 5637 cells were performed as described in Materials and Methods and assessed after 16 hours of IGF-I stimulation. Values are expressed as fold change over SFM and represent mean ± SD. *P = 0.046. (*D*) FAK-depleted 5637 cells were tested for Akt and MAPK activation after 10 minutes of IGF-I stimulation using a mix of phospho-specific antibodies (PathScan Cocktail I). eIF4E monitors protein loads. Blot is representative of three independent experiments.

Collectively, these results do not support a critical role for FAK in regulating IGF-IR-dependent motility and invasive capability of urothelial cancer cells.

### Pyk2 is Critical for IGF-I-induced Motility, Invasion and Signaling

It is known that Pyk2 can promote both distinct and overlapping signaling events with FAK [23], [24]. As we could not establish a major role for FAK in IGF-I-evoked motility of urothelial cancer cells, we considered the alternate hypothesis that Pyk2 is a predominant intracellular kinase that could mediate the downstream signaling pathway triggered by activation of the IGF-IR in urothelial cancer cells.

First, we discovered that IGF-I stimulation of 5637 cells induced a prolonged Pyk2 activation, which was sustained for up to 2 hours, as determined by immunoblot with anti-Phospho-Pyk2 antibody (Figure 2A). Second, we performed transient transfection assays in 5637 cells and determined that overexpression of wild type Pyk2 significantly increased IGF-I-induced migration, which was inhibited by the expression of a kinase-dead dominant negative Pyk2 (**P<0.01, compared to V-transfected cells) (Figure 2B). Proper expression of Flag-tagged wild-type or kinase-dead Pyk2 proteins was determined by immunoblot with anti-Flag antibodies (Figure 2C).

**Figure 2:** IGF-I-activated Pyk2 is critical for IGF-IR-dependent motility of invasive urothelial cancer cells. (*A*) Serum-starved 5637 cells were stimulated with 50 ng/ml of IGF-I for the indicated time points. Pyk2 phosphorylation was detected by immunoblot using anti-phospho-Pyk2 (Tyr402) antibodies, while total Pyk2 protein level was assessed using anti-Pyk2 polyclonal antibodies. Blot is representative of two independent experiments. (*B*) Migration of 5637 cells transiently transfected with either Flag-tagged wild type (PYK2 WT) or a dominant negative (KD PYK2) Pyk2 proteins was assessed after 16 hours of IGF-I stimulation. Values are expressed as fold change over SFM and represent mean ± SD. ** *P*<0.01. (*C*) Expression levels of transiently transfected Pyk2 proteins were assessed by immunoblot with anti-flag M2 antibodies. Blot is representative of two independent experiments.

Next, to confirm Pyk2 function, we depleted endogenous Pyk2 in 5637 cells by siRNA approaches. Pyk2 depletion (Figure 3A) severely inhibited IGF-I-induced tumor cell migration (Figure 3B) and invasion through Matrigel™ (Figure 3C). Interestingly, Pyk2 depletion slightly upregulated FAK levels (Figure 3A), although FAK was unable to compensate for Pyk2 loss. In addition, Pyk2 knockdown in 5637 cells affected IGF-IR-downstream signaling and inhibited IGF-I-dependent activation of Akt and ERK1/2 and downstream effectors S6K and p90RSK (Figure 3D).

**Figure 3:** Pyk2 is critical for IGF-IR-induced motility, invasion and signaling of invasive urothelial cancer cells. (A) 5637 cells were transfected with the Pyk2 siGenome pool or control. After 72 hours Pyk2 and FAK expression was detected by immunoblot with specific antibodies. Blot is representative of three independent experiments with an average Pyk2 depletion level of 92.6±3 (arbitrary units) as assessed by densitometric analysis (B and C) Migration and invasion of 5637 cells were assessed as described in Materials and Methods after 16 hours of IGF-I stimulation. Values are expressed as fold change over SFM and represent mean ± SD. *P<0.05; **P<0.01. (*D*) Pyk2-depleted 5637 cells were tested for the activation of the Akt and MAPK pathways after 10 min of IGF-I stimulation using a mix of phospho-specific antibodies (PathScan Cocktail I). eIF4E monitors protein loads. Blot is representative of three independent experiments.

To corroborate our results on Pyk2 function, we transiently depleted by siRNA approaches endogenous Pyk2 in T24 cells, another IGF-I-responsive invasive urothelial cancer cell line [17], [18]. We achieved a significant reduction in Pyk2 levels (Figure S1A) with a concurrent reduction in the ability of T24 cells to migrate (Figure S1B) and invade (Figure S1C) in response to IGF-I stimulation (*P<0.05, compared to either mock transfected or control oligo-transfected cells). In addition, Pyk2 ablation in T24 cells was associated with reduced IGF-I-dependent activation of ERK1/2 and S6K, while Akt and p90RSK activation was not affected (Figure S1D).

Collectively, our findings reveal an essential role for Pyk2 in the IGF-IR functional regulation of tumor cell motility and invasion, key properties of the aggressive cancer phenotype.

### Pyk2 colocalizes with the IGF-IR and Complexes with IRS-1/2 and Grb2 in Urothelial Cancer Cells

To determine whether Pyk2 may interact with the IGF-IR in 5637 cells, we initially performed co-immunoprecipitation assays but we were unable to detect an interaction between endogenous IGF-IR and Pyk2 proteins. Thus, we used confocal microscopy analysis to determine whether Pyk2 may colocalize with the IGF-IR in 5637 urothelial cancer cells. While in serum-starved 5637 cells Pyk2 did not colocalize with the IGF-IR (Figure 4A), 30 minutes of IGF-I stimulation induced significant colocalization of endogenous Pyk2 and IGF-IR proteins (Figure 4A) suggesting that Pyk2 may be recruited to the IGF-IR upon ligand stimulation.

**Figure 4:** Pyk2 colocalizes with the IGF-IR and complexes with IRS-2 and Grb2 after IGF-I stimulation of urothelial cancer cells. (A) 5637 cells were serum-starved over night and then treated with 50 ng/ml of IGF-I for 30 minutes. After fixation, cells were labeled with a monoclonal anti-IGF-IR (green) and a polyclonal anti-Pyk2 (red) and imaged by confocal microscopy. The pictures of merged fields show colocalization (yellow) of IGF-IR and Pyk2 in the IGF-I treated cells (arrows) but not in unstimulated control cells. The distinct co-localization of Pyk2 and IGF-IR is detectable in the Z stacks (yellow staining, bottom panel). Pictures are representative of at least 10 independent fields from two independent experiments. An average of 300 cells was examined for each condition. Bar: 10 µm. (B) 5637 and(C) T24 bladder cancer cells were serum-starved for 24 hours and then stimulated with 50 ng/ml of IGF-I for 30 minutes. Two mg of cell lysates were immunoprecipitated with anti-Pyk2 polyclonal antibodies. IRS-1, IRS-2, Grb2 and Pyk2 levels were assessed by immunoblot with specific polyclonal antibodies. Blots are representatives of three independent experiments.

Next, to investigate the mechanisms by which Pyk2 regulates IGF-IR downstream signaling, we performed co-immunoprecipitation assays in both 5637 and T24 cells. The main goal of these studies was to determine whether Pyk2 would complex with the docking proteins IRS-1 and/or IRS-2 or Grb2 adaptors, known to regulate IGF-IR-dependent activation of the Akt and MAPK pathways, respectively [25], [26], [27]. In 5637 cells, IRS-1 was detectable in complex with Pyk2 in unstimulated cells but uncoupled from Pyk2 after 30 minutes of IGF-I stimulation (Figure 4B). In contrast, IRS-2 binding to Pyk2 was barely detectable in serum-starved 5637 cells but strongly increased after IGF-I stimulation (Figure 4B). Grb2 recruitment to Pyk2 was detectable in unstimulated 5637 cells but it was strongly enhanced after ligand stimulation (Figure 4B). The same results were recapitulated in T24 cells with only some differences in the levels of IRS-1, IRS-2 and Grb2 detectable in Pyk2 co-immunoprecipitates (Figure 4C). These qualitative differences may be likely due to differences in the relative abundance of these proteins in 5637 and T24 cells as in fact 5637 cells express higher level of Pyk2 proteins compared to T4 (data not shown). In addition, the interaction between Pyk2, IRS-1 and IRS-2 could be indirect and mediated by additional associated proteins, which may differ between 5637 and T24 cells.

These results indicate that Pyk2, by recruiting IRS-2 and Grb2, could play a critical role in regulating IGF-IR-dependent activation of downstream signaling pathways required for motility and invasion of urothelial cancer cells.

### Pyk2 is Overexpressed in Bladder Cancer Tissues

We have recently shown that the IGF-IR is overexpressed in invasive bladder cancer tissues compared to normal tissue controls [17] and IGF-IR levels increase with bladder cancer progression [18]. Thus, we determined the expression of Pyk2 in a well annotated bladder cancer tissue microarray using immunofluorescence and AQUA analysis (Automated Quantitative Analysis) [28]. Pyk2 expression significantly increased in various bladder cancer tissues types (Figure 5A and B) as compared to normal tissue controls. In addition, the AQUA analysis for Pyk2 expression in various cellular compartments revealed that there was a significantly higher level of Pyk2 expression in the nuclei of urothelial cancer tissue cells when compared to cells in normal tissues (*P = 0.012, Figure 5C).

**Figure 5:** Pyk2 is up-regulated in bladder cancer tissues. (A) Pyk2 expression on a bladder cancer tissue microarray was determined by immunofluorescence and AQUA analysis using the AQUA PM-2000 system (HistoRx, Inc). Automated quantification and statistics on the different types of bladder cancer tumor tissues (B) and in the cytoplasmic and nuclear fractions of urothelial carcinoma cells (C) was calculated by AQUA Software. (B) *P<0.05. **P<0.01 compared to normal tissue controls. (C) *P = 0.012 compared to non-neoplastic nuclear fraction.

Nuclear Pyk2 staining is better visualized at higher magnification of selected field of normal and urothelial carcinoma tissues (Figure S2).

Collectively, our results have identified a novel protein in the IGF-IR pathway that may be critical for bladder cancer. They also provide the first evidence that Pyk2 may translocate into the nuclei of bladder cancer cells. In addition, Pyk2 may serve in conjunction with the IGF-IR as a novel diagnostic and possibly prognostic biomarker for bladder cancer.

## Discussion

The molecular mechanisms that determine malignant transformation of urothelial cells in the bladder are still very poorly characterized. In addition, there is an urgent need to identify proteins that may play a key role in driving the progression to the invasive and possibly metastatic phenotype in bladder neoplasia [2], [3], [4].

We have recently established that activation of the IGF-IR does not evoke *in vitro* cell proliferation but promotes motility and invasion of urothelial cancer cells [17], [18]. These results support the hypothesis that the IGF-IR may not be so critical for bladder cancer initiation, but may play a prominent role during progression to the invasive and possibly metastatic stage of bladder cancer.

Based on our previous observation that upon IGF-I-stimulation FAK localizes with paxillin at dynamic adhesion sites of migrating cells [17], we investigated whether FAK, or its homolog Pyk2, would modulate IGF-IR action in urothelial cancer cells. We demonstrate that: (i) Depletion of endogenous FAK protein by siRNA strategies does not affect IGF-I-dependent motility and signaling of 5637 urothelial cancer cells. (ii) The FAK homolog Pyk2 is activated upon IGF-I stimulation of 5637 cells. (iii) Transient expression of wild type Pyk2 enhances IGF-I-induced migration, which is severely inhibited instead by the expression of a dominant-negative kinase-dead Pyk2 mutant. (iv) Pyk2 depletion by siRNA approaches inhibits IGF-I-dependent migration and invasive ability of 5637 and T24 cells and affects IGF-IR downstream signaling. (v) Upon IGF-I stimulation Pyk2 complex with IRS-2 and Grb2 in 5637 and T24 urothelial cancer cells. (vi) Pyk2 is overexpressed in various bladder cancer tissue types compared to normal tissue controls. (vii) Pyk2 expression increases in the nuclei of urothelial cancer tissue cells compared to normal tissue cells.

FAK and Pyk2 are related tyrosine-kinases involved in the dynamic regulation of the actin cytoskeleton, a process critical for cell motility, mitosis and tumor progression [24], [29]. FAK and Pyk2 share a conserved molecular architecture and exhibit an overall 45% sequence identity with the greatest sequence identity (60%) in the kinase domain [24], [29]. FAK is ubiquitously expressed while Pyk2 expression has a more limited tissue distribution with the highest Pyk2 expression levels detected in cells of the central nervous system and in hematopoietic lineage [29]. In addition, FAK and Pyk2 differs for their intracellular distribution, with FAK prevalently expressed at focal adhesions while Pyk2 expression is more distributed throughout the cell and sometimes enriched in perinuclear regions [29].

We have recently shown that IGF-I stimulation of invasive urothelial cells induces paxillin phosphorylation at Tyrosine 31 [17], a process mediated by FAK in other cellular models [21]. We further showed that paxillin localizes with FAK at the leading edge of migrating cells [17]. Because in other tumor models FAK is required for PI3K- and Ras-dependent tumorigenesis [30] and the integrins/FAK complex activates Ras signaling to MAPK [31], [32] a plausible mechanism by which IGF-I promotes migration and invasion of bladder cancer cells would be by activating FAK and the signaling cascade leading to Akt, MAPK and paxillin activation. Surprisingly, FAK depletion in 5637 cells had no effect in modulating both IGF-I-induced migration and IGF-IR-dependent activation of the Akt and MAPK pathways. The modest inhibitory effect on invasion detected in FAK-depleted 5637 cells in the absence of MAPK and Akt inhibition suggest that additional MAPK- and Akt-independent pathways may partially contribute to FAK-dependent invasive signaling in these cells.

However, we discovered that altering Pyk2 expression by transient overexpression of either wild type or dominant-negative Pyk2 proteins, or by siRNA-mediated Pyk2 depletion, had a major effect on IGF-I-induced motility and invasive ability of 5637 and T24 urothelial cancer cells. These functional assays were further corroborated by biochemical assays showing a significant inhibition of IGF-IR-activation of downstream signaling when intracellular Pyk2 levels were reduced. Thus, these results suggest that Pyk2 may have a more prevalent role than FAK in regulating IGF-IR-dependent biological responses in invasive urothelial cancer cells.

As Pyk2 depletion severely inhibits IGF-I-induced signaling, it could be argued that the effects of Pyk suppression on migration are a consequence of reduced proliferation/survival. However, we have previously shown that in both 5637 and T24 urothelial cancer cells the ability of IGF-I to induce motility (migration and invasion) is totally independent from the IGF-IR ability to sustain proliferation/survival, as in fact IGF-I does not enhance cell growth in these cells, which proliferate in the absence of serum [17].

To investigate the mechanisms by which Pyk2 may regulate IGF-I-dependent biological responses in urothelial cells, we initially assessed by confocal microscopy whether upon IGF-I-stimulation Pyk2 colocalized with paxillin in focal adhesions. However, in both serum-starved and IGF-I-stimulated 5637 and T24 cells we could not detect any colocalization of Pyk2 and paxillin, and Pyk2 staining was more diffuse throughout the cytoplasm and not enriched in focal adhesions (not shown). In addition, we performed co-immunoprepitation experiments in which we failed to detect a Pyk2/paxillin complex (not shown). These results strongly indicate that Pyk2 action in regulating IGF-I-dependent motility of urothelial cancer cells can be separated from paxillin function at focal adhesions.

Ligand-dependent recruitment of IRS-1/2 and Grb2 proteins to the IGF-IR is a critical step in the activation of the Akt and MAPK pathways in various IGF-IR-dependent biological responses [25], [33], [34], [35], [36]. Interestingly, IGF-I stimulation of 5637 and T24 urothelial cancer cells evoked the formation of a complex containing Pyk2, IRS-2 and Grb2 suggesting that in urothelial cancer cells Pyk2 may work as a critical signaling hub downstream of the IGF-IR. Whether Pyk2 binds directly to the IGF-IR and mediates the recruitment of IRS-2 and Grb2 to the receptor has not been demonstrated. So far we have not being able to detect an interaction between the IGF-IR and Pyk2 by co-immunoprecipitation experiments in 5637 cells but this negative result could be likely attributed to the relative low level of endogenous proteins. On the other hand, this result could also indicate that the IGF-IR and Pyk2 may interact indirectly in a complex with other signaling molecules of the IGF-IR system, such as IRS-1 and IRS-2. However, we have demonstrated by confocal microscopy that the IGF-IR and Pyk2 colocalize in ligand-dependent fashion suggesting that Pyk2 upon IGF-I stimulation may complex with the IGF-IR and facilitate the recruitment of signaling molecules to the receptor.

Recent experiments in vascular smooth muscle cells have demonstrated that upon IGF-I stimulation Pyk2 mediates the recruitment of Grb2 to the signaling SHP-1/SHP2/Src complex thus promoting MAPK activation and cell proliferation [37]. However, whether a similar mechanism may be conserved in urothelial cancer cells remains to be elucidated.

Our recent data have demonstrated that the IGF-IR is overexpressed in invasive bladder cancer tissues compared to normal tissue controls [17] and IGF-IR levels increase with bladder cancer progression [18]. The AQUA analysis we performed shows that Pyk2 expression is significantly upregulated in various bladder cancer tissue subtypes compared to normal controls but we could not detect a statistically significant difference in Pyk2 expression levels associated with different stages of urothelial carcinoma. A study with a larger sampling representing different stages of urothelial carcinoma is required to clearly establish whether Pyk2 may work as a prognostic marker for bladder cancer progression. Interestingly, in urothelial carcinoma cells the AQUA analysis revealed a statistically significant increase in the fraction of Pyk2 detected in the nucleus compared to cells in normal controls. Pyk2 localization in the nucleus has been previously demonstrated [38], [39] but the function of Pyk2 in the nucleus has not been characterized. Our results provide the first evidence of increased levels of nuclear Pyk2 in bladder cancer cells thereby suggesting the novel hypothesis that in bladder cancer cells IGF-I-activated Pyk2 may act not only in the cytoplasm but also translocate into the nucleus, where it might work as a transcription factor. Significantly, IRS-1 and IRS-2 proteins have been shown to translocate to the nucleus in several cancer cell models [40], [41], [42], [43], where they regulate gene expression [43], [44]. In addition IRS-1 level in the nucleus predicts tamoxifen response in patients with early breast cancer [45], Thus, our results suggest the attractive hypothesis that IRS-1 or IRS-2 proteins may play a role in regulating Pyk2 translocation and/or interact with Pyk2 in the nucleus.

Experiments are currently under way to determine whether Pyk2 nuclear translocation is detectable in various urothelial cancer cell lines and is mediated by IGF-I. Future experiments will also determine IRS-1 or IRS-2 action in regulating Pyk2 nuclear translocation and function.

In conclusion, we have identified Pyk2 as a novel critical regulator of IGF-IR-dependent motility and invasion of urothelial cancer cells. These studies will greatly contribute to the identification of novel targets for therapeutic intervention in bladder tumors. In addition IGF-IR and Pyk2 may work as novel biological markers for bladder cancer progression.

## Materials and Methods

### Cells and Materials

Urothelial carcinoma-derived human 5637 and T24 cells were obtained from ATCC (Manassas, VA, USA. 5637 and T24 cells were maintained in RPMI medium supplemented with 10% fetal bovine serum (FBS). Serum-free medium (SFM) is DMEM supplemented with 0.1% bovine serum albumin and 50 µg/mL of transferrin (Sigma-Aldrich, St Louis, MO, USA). Recombinant IGF-I was purchased from Calbiochem (San Diego, CA, USA).

### siRNA-mediated Gene Silencing

To silence FAK or Pyk2 we used RNA interference by using small-interfering RNA (siRNA). 5637 and T24 cells were transfected with vehicle (DEPC-treated water), control siRNA (scrambled), or siRNA specific oligos (200–400 pmol/L) using the TransIT-siTKO reagent (Mirus Bio LLC, Madison, WI, USA). Both scrambled and anti-FAK or anti-PYK2 siRNA oligos were from Thermo Scientific Dharmacon (siGenome Smartpool siRNA) (Lafayette, CO, USA). Cells were analyzed for motility and signaling 72 hours post-transfection. siRNA efficiency was detected by immunobloting using anti-FAK (#3285) and anti-Pyk2 (#3090) polyclonal antibodies (both from Cell Signaling Technology, Beverly, MA, USA). ß-actin was detected using anti-ß-actin polyclonal antibody (Sigma-Aldrich). Densitometric analysis was performed using the ImageJ program (rsbweb.nih.gov/ij/).

### Transient Transfection Assays

5637 cells were transiently transfected using the TransIT®-Prostate Transfection Kit (Mirus BIO LLC) with the expression plasmid pShCMV.3X FLAG expressing either wild type or kinase-dead (K457A) Pyk2 mutant protein. Forty-eight hours post transfection, cells were serum-starved for additional 24 hours and then stimulated or not with 50 ng/mL of IGF-I. Migration was determined after 18 hours of incubation with the ligand, as stated below. In parallel, cells were lysed with cold RIPA buffer and the expression of the transfected plasmids was detected by western blot analyses using an anti-FLAG antibody (Santa Cruz Biotechnologies, Inc.).

### Migration and Invasion Assays

5637 or T24 cells were plated in duplicate at a density of 3×10^4^ cells/35-mm^2^ plates in serum-supplemented medium. After 24 hours, cells were transferred to SFM or SFM supplemented with 50 ng/mL of IGF-I. Migration or invasion experiments were carried on for 4 hours or 16 hours, depending on the cell line used (T24 or 5637, respectively). Migration experiments were performed using HTS FluoroBloks™ inserts (BD, San Jose, CA, USA) as previously described [17], [18], [46], [47]. Membranes were mounted on a slide and migrated cells were counted and photographed with a Zeiss Axiovert 200 M cell live microscope at the Kimmel Cancer Center Bioimaging Facility. Cell invasion through a 3D-extracellular matrix was assessed using BD Matrigel™-coated Invasion Chambers (BD Biocoat) [17], [18], [47]. After 24 hours filters were washed, fixed, and stained with Coomassie Brilliant Blue. Cells that had invaded to the lower surface of the filter were counted under the microscope.

### Analyses of Protein/Protein Interactions

5637 or T24 cells were serum-starved for 24 hours and then stimulated with IGF-I (50 ng/mL) for 30 minutes. Cells were lysed in cold RIPA buffer without sodium deoxycholate. The insoluble material was separated by centrifugation and the supernatants were incubated at 4°C under rotation for 18 hours with anti-Pyk2 polyclonal antibody (Sigma-Aldrich). At the end of the incubation, immunocomplexes were separated by adding 30 µL of mix protein A/G-Sepharose for additional 30 minutes. The resolved proteins were reduced in 40 µL of Laemmli buffer and subjected to SDS-PAGE. IRS-1 and IRS-2 interactions were determined by immunoblot using Anti-IRS-1 and Anti-IRS-2 polyclonal antibodies from Millipore (Burlington, MA, USA). The anti-Grb2 monoclonal antibody is from BD Biosciences. Blots are representative of three independent experiments.

### Detection of Activated Signaling Pathways

5637 or T24 cells were serum-starved for 24 hours and then stimulated with IGF-I (50 ng/mL) for 5, 10, 30 and 120 minutes. Pyk2 phosphorylation was detected by immunoblot using anti-phospho-Pyk2 (Tyr-402) antibodies (Cell Signaling Technology). The activation of p90RSK, Akt, ERK1/2 and S6 Ribosomal Protein was analyzed by western immunoblot using the PathScan Multiplex Western Cocktail I (Cell Signaling Technology). ElF4E protein is used as control to monitor the loading of the samples.

### Confocal Microscopy

5637 cells were plated onto 4-well chamber slides (BD Bioscences) and serum-starved over night prior to treatment with 50 ng/ml of IGF-I for 10, 30 and 60 minutes. Cells were then washed with 1X PBS and fixed with 4% PFA for 30 minutes at room temperature. Subsequently, slides were subjected to immunofluorescence and confocal analysis as previously described [18], [46], [48], [49], [50]. Primary antibodies were anti-IGF-IR monoclonal (Calbiochem) and anti-Pyk2 polyclonal antibodies (Santa Cruz Biotechnologies). Secondary antibodies were goat anti-mouse IgG Alexa Fluor® 488 and goat anti-rabbit IgG Alexa Fluor® 594 antibodies (Invitrogen). Confocal analysis was performed on a Zeiss LSM810 microscope. The filters were set to 488 and 594 nm for dual channel imaging. All the images were then analyzed using Image J and Adobe Photoshop CS3 (Adobe Systems, San Jose, CA) software.

### Pyk2 Expression in Bladder Cancer Tissues

Pyk2 expression levels in bladder cancer tissue were determined by AQUA analysis (Automated Quantitative Analysis) [28] on an Accumax bladder cancer tissue microarray (TMA #A215), composed by 4 non neoplastic spots and 45 different bladder cancer tissues (n = 33 urothelial carcinoma, n = 5 adenocarcinoma, n = 4 squamous carcinoma and n = 3 urothelial carcinoma in situ, two spots for each case). Detailed information regarding the TMA used is available on Accumax website. The antibodies used for immunofluorescence were rabbit pan-cytokeratin antibody (Cy2 conjugated, DAKO), Pyk2 antibody (Rabbit monoclonal YE353, Abcam) and DAPI. Pyk2 antibody was conjugated with Cy5 since it is outside the auto-fluorescence spectrum of tissue. Nuclear and cytoplasmic mask were automatically defined by AQUA Software, and applied to quantify Pyk2 expression on TMA. The analysis was performed at the Kimmel Cancer Center Translational Core Facility using an AQUA PM-2000 system (HistoRx, Inc). Automated quantification and statistics was calculated by AQUA Software. *P<0.05. **P<0.01 compared to normal.

### Statistical Analysis

Experiments were carried out in triplicate and repeated at least three times. Results are expressed as mean ± SD. All statistical analyses were carried out with PRISM GraphPad Software, v.5. Results were compared using the two-sided Student’s t test. Differences were considered statistically significant at *P*<0.05.

## Supporting Information

Figure S1 **Pyk2 is critical for IGF-IR-induced motility, invasion and signaling of invasive urothelial cancer cells. (**A) T24 cells were transfected with the Pyk2 siGenome pool or control. After 72 hours Pyk2 and FAK expression was detected by immunoblot with specific antibodies. Blot is representative of three independent experiments with an average Pyk2 depletion level of 93.4±3.5 (arbitrary units) as assessed by densitometric analysis (B and C) Migration and invasion of T24 cells were assessed as described in Materials and Methods after 4 hours of IGF-I stimulation. Values are expressed as fold change over SFM and represent mean ± SD. *P<0.05. (D) Pyk2-depleted T24 cells were tested for the activation of the Akt and MAPK pathways after 10 min of IGF-I stimulation using a mix of phosphor-specific antibodies (Pathscan cocktail I). eIF4E monitors protein loads. Blot is representative of three independent experiments.
(TIF)

Figure S2 **Pyk2 is up-regulated in urothelial carcinoma.** Pyk2 expression on a bladder cancer tissue microarray was determined by immunofluorescence and AQUA analysis using the AQUA PM-2000 system (HistoRx, Inc). Higher magnification images from the same normal and urothelial carcinoma tissue samples shown in Figure 5 were acquired using a LEICA DM5500B microscope equipped with Leica Application Suite, Advanced Fluorescence 1.8 software (Leica Mycrosystem, Inc.) using a 63X Objective. Pictures are representative of at least 10 independent fields. Bar ∼10 µm.
(TIF)

## References

[1] Siegel R, Naishadham D, Jemal A (2012). Cancer statistics, 2012.. CA: A Cancer Journal for Clinicians.

[2] Mitra AP, Cote RJ (2009). Molecular Pathogenesis and Diagnostics of Bladder Cancer.. Annu Rev Pathol.

[3] Knowles MA (2008). Molecular pathogenesis of bladder cancer.. Int J Clin Oncol.

[4] Goebell PJ, Knowles MA (2010). Bladder cancer or bladder cancers? Genetically distinct malignant conditions of the urothelium.. Urol Oncol.

[5] Scher CD, Stone ME, Stiles CD (1979). Platelet-derived growth factor prevents G0 growth arrest.. Nature.

[6] Baserga R (1995). The insulin-like growth factor I receptor: a key to tumor growth?. Cancer Res.

[7] Baker J, Liu JP, Robertson EJ, Efstratiadis A (1993). Role of insulin-like growth factors in embryonic and postnatal growth.. Cell.

[8] Eggenschwiler J, Ludwig T, Fisher P, Leighton PA, Tilghman SM (1997). Mouse mutant embryos overexpressing IGF-II exhibit phenotypic features of the Beckwith-Wiedemann and Simpson-Golabi-Behmel syndromes.. Genes Dev.

[9] Sell C, Dumenil G, Deveaud C, Miura M, Coppola D (1994). Effect of a null mutation of the insulin-like growth factor I receptor gene on growth and transformation of mouse embryo fibroblasts.. Mol Cell Biol.

[10] Surmacz E (2003). Growth factor receptors as therapeutic targets: strategies to inhibit the insulin-like growth factor I receptor.. Oncogene.

[11] Baserga R, Morrione A (1999). Differentiation and malignant transformation: two roads diverged in a wood.. J Cell Biochem.

[12] Pollak MN, Schernhammer ES, Hankinson SE (2004). Insulin-like growth factors and neoplasia.. Nat Rev Cancer.

[13] Le Roith D, Karas M, Yakar S, Qu BH, Wu Y (1999). The role of the insulin-like growth factors in cancer.. Isr Med Assoc J.

[14] Baserga R (2000). The contradictions of the insulin-like growth factor 1 receptor.. Oncogene.

[15] Baserga R, Hongo A, Rubini M, Prisco M, Valentinis B (1997). The IGF-I receptor in cell growth, transformation and apoptosis.. Biochim Biophys Acta.

[16] Le Roith D (2000). Regulation of proliferation and apoptosis by the insulin-like growth factor I receptor.. Growth Horm IGF Res 10 Suppl A.

[17] Metalli D, Lovat F, Tripodi F, Genua M, Xu SQ (2010). The insulin-like growth factor receptor I promotes motility and invasion of bladder cancer cells through Akt- and mitogen-activated protein kinase-dependent activation of paxillin.. Am J Pathol.

[18] Iozzo RV, Buraschi S, Genua M, Xu SQ, Solomides CC (2011). Decorin antagonizes IGF-IR function by interfering with IGF-IR activity and attenuating downstream signaling.. J Biol Chem.

[19] Lev S, Moreno H, Martinez R, Canoll P, Peles E (1995). Protein tyrosine kinase PYK2 involved in Ca(2+)-induced regulation of ion channel and MAP kinase functions.. Nature.

[20] Yu H, Li X, Marchetto GS, Dy R, Hunter D (1996). Activation of a novel calcium-dependent protein-tyrosine kinase. Correlation with c-Jun N-terminal kinase but not mitogen-activated protein kinase activation.. J Biol Chem.

[21] Zhao J, Guan JL (2009). Signal transduction by focal adhesion kinase in cancer.. Cancer Metastasis Rev.

[22] Webb DJ, Donais K, Whitmore LA, Thomas SM, Turner CE (2004). FAK-Src signalling through paxillin, ERK and MLCK regulates adhesion disassembly.. Nat Cell Biol.

[23] Weis SM, Lim ST, Lutu-Fuga KM, Barnes LA, Chen XL (2008). Compensatory role for Pyk2 during angiogenesis in adult mice lacking endothelial cell FAK.. J Cell Biol.

[24] Lipinsky CA, FLoftus JC (2010). The Pyk2 FERM domain: a Novel Therapeutic Target.. Expert Opin Ther Targets.

[25] Morrione A, Romano G, Navarro M, Reiss K, Valentinis B (2000). Insulin-like growth factor I receptor signaling in differentiation of neuronal H19–7 cells.. Cancer Res.

[26] Peruzzi F, Prisco M, Dews M, Salomoni P, Grassilli E (1999). Multiple signaling pathways of the insulin-like growth factor 1 receptor in protection from apoptosis.. Mol Cell Biol.

[27] Peruzzi F, Prisco M, Morrione A, Valentinis B, Baserga R (2001). Anti-apoptotic signaling of the insulin-like growth factor-I receptor through mitochondrial translocation of c-Raf and Nedd4.. J Biol Chem.

[28] Rubin MA, Zerkowski MP, Camp RL, Kuefer R, Hofer MD (2004). Quantitative determination of expression of the prostate cancer protein alpha-methylacyl-CoA racemase using automated quantitative analysis (AQUA): a novel paradigm for automated and continuous biomarker measurements.. Am J Pathol.

[29] Schaller MD (2010). Cellular functions of FAK kinases: insight into molecular mechanisms and novel functions.. J Cell Sci.

[30] Pylayeva Y, Gillen KM, Gerald W, Beggs HE, Reichardt LF (2009). Ras- and PI3K-dependent breast tumorigenesis in mice and humans requires focal adhesion kinase signaling.. J Clin Invest.

[31] Guo W, Giancotti FG (2004). Integrin signalling during tumour progression.. Nat Rev Mol Cell Biol.

[32] Bao W, Stromblad S (2004). Integrin alphav-mediated inactivation of p53 controls a MEK1-dependent melanoma cell survival pathway in three-dimensional collagen.. J Cell Biol.

[33] Valentinis B, Romano G, Peruzzi F, Morrione A, Prisco M (1999). Growth and differentiation signals by the insulin-like growth factor 1 receptor in hemopoietic cells are mediated through different pathways.. J Biol Chem.

[34] Valentinis B, Navarro M, Zanocco-Marani T, Edmonds P, McCormick J (2000). Insulin receptor substrate-1, p70S6K, and cell size in transformation and differentiation of hemopoietic cells.. J Biol Chem.

[35] Morrione A, Navarro M, Romano G, Dews M, Reiss K (2001). The role of the insulin receptor substrate-1 in the differentiation of rat hippocampal neuronal cells.. Oncogene.

[36] Dews M, Prisco M, Peruzzi F, Romano G, Morrione A (2000). Domains of the insulin-like growth factor I receptor required for the activation of extracellular signal-regulated kinases.. Endocrinology.

[37] Shen X, Xi G, Radhakrishnan Y, Clemmons DR (2010). Recruitment of Pyk2 to SHPS-1 signaling complex is required for IGF-I-dependent mitogenic signaling in vascular smooth muscle cells.. Cell Mol Life Sci.

[38] Farshori PQ, Shah BH, Arora KK, Martinez-Fuentes A, Catt KJ (2003). Activation and nuclear translocation of PKCdelta, Pyk2 and ERK1/2 by gonadotropin releasing hormone in HEK293 cells.. J Steroid Biochem.

[39] Aoto H, Sasaki H, Ishino M, Sasaki T (2002). Nuclear translocation of cell adhesion kinase beta/proline-rich tyrosine kinase 2.. Cell Struct Funct.

[40] Lassak A, Del Valle L, Peruzzi F, Wang JY, Enam S (2002). Insulin receptor substrate 1 translocation to the nucleus by the human JC virus T-antigen.. J Biol Chem.

[41] Wu A, Sciacca L, Baserga R (2003). Nuclear translocation of insulin receptor substrate-1 by the insulin receptor in mouse embryo fibroblasts.. Journal of Cellular Physiology.

[42] Sun H, Tu X, Prisco M, Wu A, Casiburi I (2003). Insulin-like growth factor I receptor signaling and nuclear translocation of insulin receptor substrates 1 and 2.. Molecular Endocrinology.

[43] Reiss K, Del Valle L, Lassak A, Trojanek J (2011). Nuclear IRS-1 and cancer.. J Cell Physiol.

[44] Wu A, Chen J, Baserga R (2008). Nuclear insulin receptor substrate-1 activates promoters of cell cycle progression genes.. Oncogene.

[45] Migliaccio I, Wu MF, Gutierrez C, Malorni L, Mohsin SK (2010). Nuclear IRS-1 predicts tamoxifen response in patients with early breast cancer.. Breast Cancer Res Treat.

[46] Monami G, Emiliozzi V, Bitto A, Lovat F, Xu SQ (2009). Proepithelin regulates prostate cancer cell biology by promoting cell growth, migration, and anchorage-independent growth.. Am J Pathol.

[47] Lovat F, Bitto A, Xu SQ, Fassan M, Goldoni S (2009). Proepithelin is an autocrine growth factor for bladder cancer.. Carcinogenesis.

[48] Monami G, Emiliozzi V, Morrione A (2008). Grb10/Nedd4-mediated multiubiquitination of the insulin-like growth factor receptor regulates receptor internalization.. J Cell Physiol.

[49] Monami G, Gonzalez EM, Hellman M, Gomella LG, Baffa R (2006). Proepithelin promotes migration and invasion of 5637 bladder cancer cells through the activation of ERK1/2 and the formation of a paxillin/FAK/ERK complex.. Cancer Res.

[50] Buraschi S, Pal N, Tyler-Rubinstein N, Owens RT, Neill T (2010). Decorin antagonizes Met receptor activity and down-regulates {beta}-catenin and Myc levels.. J Biol Chem.

